# Research on Information Leakage Tracking Algorithms in Online Social Networks

**DOI:** 10.1155/2022/5634385

**Published:** 2022-10-04

**Authors:** Junli Xiong, Huayi Huang

**Affiliations:** ^1^Computer Engineering Technical College (Artificial Intelligence College), GuangDong Polytechnic of Science and Technology, ZhuHai 519090, China; ^2^School of Computer Science, South China Normal University, GuangZhou 510000, China

## Abstract

An online social network is a platform where people can communicate with friends, share information, speed up business development, and improve teamwork. A large amount of user privacy information existing in real social networks is leaked from person to person, and this issue has hardly been studied. With the rapid expansion of the network, the issue of privacy protection has received increasing attention. So far, many privacy protection methods including differential protection algorithms, encryption algorithms, access control strategies, and anonymization have been researched and applied. Information leakage means that the information shared by the user is disseminated or downloaded by his friends without the user's consent, and the transmission of private information will not be recorded. In order to track and find out the ways and methods of information leakage, this article adopts an unusual method, namely, the probability judgment based on trust. By screening the similarities between users, past information exchanges, and the topology of social networks, a trust model is established to evaluate and estimate the degree of trust between users. According to the rating information privacy of friends' trust, an information dissemination system is established, which can be applied to online social networking platforms to reduce the risk of information leakage, thereby ensuring the security of users' private information. At the same time, this paper expands the transmission system model without user authorization and proposes a fingerprint-based deterministic leak tracking algorithm.

## 1. Introduction

At present, the registration of various software requires the entry of personal information, including private information such as identity information, social relations, and financial transaction information, and the purpose of submitting user-related data information is to confirm the authenticity of their identity information, for example, the current implementation The real-name system is to ensure that users experience it personally, and each step is operated by themselves [1, 2]. And it is precisely this kind of operation that was originally believed to be safe to leak users' information, making the interests of online social network users unable to be protected, as if they may be stolen at any time, and it is urgent to use technological means to protect their interests [3]. However, the research focus of traditional social networks is to protect big data from infringement, and common information leakage methods are not mentioned. Often such violations of privacy cannot be confirmed on social media, and it is difficult to find the source of information leakage [4]. For example, if an individual leaks a secret to another individual and this secret subsequently appears on other platforms, then the culprit of the leaked information is obvious and beyond doubt. But, if multiple people know this secret at the same time, things will become very complicated [5]. Assuming that everyone gets the exact same data at the same time and one of them secretly leaked the secret, it is mathematically impossible to determine whether a person is guilty or not. Therefore, it can be considered that when some people have all the data, but others do not, then the security of the information can be improved by encrypting the data [6]. When many customers purchase digital rights, data providers provide customers with keys so that they can unlock the encrypted data. However, it is generally believed that the encryption method cannot solve the fundamental problem because it cannot prevent the authorization to view the message while sending it out, and it is impossible to view the downloading of the information and the purpose of the information. This way of disseminating and disclosing information is also impossible to trace the source. We call it unauthorized verbal errors [7]. It is this kind of human-to-human verbal error that has brought unimaginable problems to our research on information leakage algorithms. Therefore, on social networking platforms, the relevant laws used by users should be clarified, that is, no one can spread the information of others by any means for any reason without the permission of others [8].

## 2. Related Work

Literature proposed a space-based text fingerprinting algorithm, which uses the word spacing of text lines to watermark text documents [9]. The coding technology adjusts the word spacing in the text document so that the average spacing between the lines shows the characteristics of the sine wave, so as to complete the sine wave coding of the information. The watermark is embedded in the horizontal and vertical directions, which has the effect of anti-interference [10]. In addition, the presence or absence of the original image does not affect the recovery of information. Literature analyzes the collusion resistance of the system to the average collusion attack, obtains performance indicators expressed in false negative probability and false positive probability, and derives the upper and lower limits of the maximum number of confluences that can meet the requirements. It is also proved that the detectors used are robust to collusion attacks of different performance [11]. Literature unknowingly inserts it into the low-frequency component of the data by spread spectrum, constructing the watermark into an independent uniform Gaussian random vector and Gaussian flux [12]. Estun introduced a two-layer codeword structure in the code domain to resist high-probability colluders. Literature proposed some digital fingerprint encoding methods for social networks, including tree structure and neighbor hashing. The literature concluded that “out-of-quantity” employees usually have a higher level of the trust relationship and the trust level of members will increase [13]. This paper proposes a trust model based on the degree of trust between online social network users. Existing trust research focuses on strange users, and the premise is that the trust of neighbor users is known. In most social network platforms, the degree of understanding between people is very low. Only through text communication to understand each other, it is impossible to fully understand each other's personality, which leads to mutual understanding of each other on social network platforms [14]. The degree of trust is greatly reduced, so in order to complete this known premise, it is necessary to evaluate the trust between adjacent users. The calculation of user familiarity not only considers the historical interaction frequency between users but also considers the number of mutual friends and the number of public communities. In the system model used this time, there are not only the data related to the network structure but also the user's past communication information on the social network platform. The system model can achieve the diversification of the use of dimensions and also ensure the comprehensiveness and accuracy of evaluation results [15], but the system model of this information leakage algorithm research is not particularly comprehensive, and the degree of research is also limited, so we need a method that enables us to use the existing data and understanding of the network structure to help us. The trust model is quantified, and the influence of the two factors is increased so that the system model can be improved.

## 3. Related Theoretical Foundations of Privacy Protection Algorithms in Social Networks

### 3.1. Social Network Model

Social networks are actually composed of two important parameters: nodes (user attributes) and their links (user interaction history). The content of the link is defined by the node according to its theme, interest, and so on (e.g., trade financing, relatives and friends, hobbies, business trade).  Figure 1 is a diagram of common social network topology. The social network itself has many characteristics. F is the collection of nodes in the social network, and the fifth is the collection of all social relations. In social networking platforms, a small number of users have more adjacent nodes, which are called central nodes. This node and a large number of nodes around it form a star network structure, as shown in Figure 1.

Online social networks are not only an opportunity but also some risks, such as the theft of users' identity information such as photos or users' messages. For solving these problems, relevant personnel have conducted relevant research and developed corresponding tools to help users better prevent privacy leakage. However, these suggestions still lack a conceptual model, which was first proposed by Aclice et al. The core is equivalent to a framework that weighs more on the privacy risks of social network users. The framework controls the mechanism from the structural attributes and outlines of the social graph to access the relationship. The most typical method is to establish a simulated trust mechanism. Through data information such as user credibility and user interaction, a dynamic trust model is established to protect user privacy and help users make decisions. This paper proposes a hybrid trust model to describe how two users trust each other. This model not only considers the direct and indirect trust between two users but also considers group trust. Trusted groups describe how users are trusted by other users in the group.

(1) The public neighbor node index is defined by the following formula:
  (1) $$\begin{array}{c} CN\left(u_{i},u_{j}\right)=\left|C\left(u_{i}\right)\cap C\left(u_{j}\right)\right|\text{.} \end{array}$$
This is the most obvious measure of trust between nodes. The more common the neighbor nodes, the higher the similarity between the two. Simply put, the more tolerant two people meet each other in social situations, the more likely they are to become friends.
(2) Jaccard index is defined by the following formula:
  (2) $$\begin{array}{c} Jaccar\;d\left(u_{i},u_{j}\right)=\frac{\left|C\left(u_{i}\right)\cap C\left(u_{j}\right)\right|}{\left|C\left(u_{i}\right)\cup C\left(u_{j}\right)\right|}\text{.} \end{array}$$
In fact, this is a way to correct the calculation of the common neighbor node index, and it is one of the factors that affect the trust value between nodes. Because in some cases, the number of public neighbors may not match the trust value between nodes.
(3) Salton index is defined by the following formula:

(3) $$\begin{array}{c} Salton\left(u_{i},u_{j}\right)=\frac{\left|C\left(u_{i}\right)\cap C\left(u_{j}\right)\right|}{\sqrt{N\left(u_{i}\right)\times N\left(u_{j}\right)}}\text{.} \end{array}$$

In summary, the three calculation methods described above are suitable for a wide range, but in addition to using the method based on the network structure to assume the trust between users, the historical interaction between users and the similarity of user attributes should also be considered.

### 3.2. Hash Mapping Algorithm

Recently, research on hashing in the fields of object retrieval, image matching, and automatic learning has attracted people's attention. Indyk et al. first studied and established the metric hash paradigm based on random projection of cosine similarity. It projects large-size data into a binary hash code and quantifies it. Hash mapping modes can be divided into two categories: independent data and dependent data.

(1) Locally sensitive hash (LSH): The basic principle of the LSH algorithm is to map similar objects (rather than distant objects) to the same storage space with high probability through a series of hash functions. Let *S* be the domain of all objects and *D* be the distance function between all objects.
  (4) $$\begin{array}{c} if\;D\left(q,p\right)\leq r,\mathrm{Pr}\;\left[h\left(q\right)=h\left(p\right)\right]\geq p_{1}\text{,}\\ ifD\left(q,p\right)\geq cr,\mathrm{Pr}\;\left[h\left(q\right)=h\left(p\right)\right]\leq p_{2}\text{.} \end{array}$$
Adjust the parameters to *c* > 1 and *p*1 > *p*2 and apply LSH to approximate the nearest neighbor search. In this regard, a type of LSH family based on hash criteria is proposed, which is defined as follows:
  (5) $$\begin{array}{c} h_{a,b}\left(v\right)=\left|\frac{\left(a*v+b\right)}{W}\right|\text{.} \end{array}$$
(2) SPH algorithm: in order to solve the random limitation of the LSH method, a machine algorithm with higher coding efficiency is used for calculation. Among them, SPH is considered to be a more effective solution, which handles the training process of the hash code of the sample data and the training process of the hash function of the data separately. We denote the incidence matrix.
  (6) $$\begin{array}{c} W\left(i,j\right)=rxp\left(\frac{-{\left\|x_{i}-x_{j}\right\|}^{2}}{\in^{2}}\right)\text{.} \end{array}$$
For in-sample data, in order to ensure that similar items can be assigned to similar code words and there are enough code words, the mapping matrix *R* of *Z* must meet the following conditions:
  (7) :YmintrYTLYs.t. yi∈−1,1k;YT1=0;YTY=1.
It is not difficult to see that the above formula is an NP-hard problem, but the vector with the smallest feature value is selected from *L*, and then these feature vectors are set aside to obtain a compromise solution, and finally, a binary code is obtained. For out-of-sample data, under the assumption that the data are uniformly distributed, a closed solution can be effectively extended to out-of-sample expansion. The specific operation method is as follows: select the PCA analysis method to find the main characteristics of *X* and use the rectangle approximate calculation along the PCA direction. The threshold value of the analysis characteristic function is reduced to zero, and the binary code is obtained. However, in the real world, it is difficult for *X* to meet the assumption of uniform data distribution, so the SPH method is not practical.
  (8) $$\begin{array}{c} W\left(i,j\right)=\left\{\begin{array}{cc} \frac{x_{i}^{T}x_{j}}{\left\|x_{i}\right\|}\cdot \left\|x_{j}\right\|\text{,} & if\;x_{i}\in N_{k}\left(x_{j}\right)\;or\;x_{j}\in N_{k}\left(x_{i}\right)\text{,}\\ 0\text{,} & otherwise\text{.} \end{array}\right. \end{array}$$
(3) STH algorithm: simply put, the principles of generating hash codes are the same for the two algorithms. In this method, a linear support vector machine (LSVM) is introduced to predict the hash code of out-of-sample data.
  (9) :w,ξi≥0min12WTW+Cn∑i=0nξi s.t:yipwTxi≥1−ξi.
Compared with SPH, the expansion of out-of-sample data in STH can ignore the assumption of uniform data distribution. However, the STH algorithm still has two important shortcomings. One is that the two-stage training method does not have the performance of the trial function when performing hash code training, resulting in poor generalization ability. Furthermore, the time cost of SVM-based classifiers in training hash codes bit by bit is immeasurable. Although the SVM classifier can be offline, it is not suitable for high-dimensional large-scale social networks.
(4) LPP algorithm: partially preserved projection: After the original data in the space is dimensionally reduced by the LPP algorithm, the relative change between the data points in the sample is not significant. At the same time, in this algorithm, after assigning an appropriate amount of weighted data points, the difference between most sample points can be enhanced, and feature matching has become more accurate and convenient. LPP is actually a linear transformation. At the same time, suppose the data set *X* = [*x*1, *x*2,…, xn], the purpose is to find a changeable matrix V and map the d-dimensional original data space to the m-dimensional data space. *Y* = [y1, y2,…, yn], where *y*_*i*_ = *V*_*xi*_ represents the data point corresponding to the low-dimensional mapping of xi. The optimized objective function is as follows:
  (10) $$\begin{array}{c} {\sum_{i,j}\left(y_{i}-y_{j}\right)}^{2}W_{ij}\text{,} \end{array}$$

where *W* is the adjacency matrix, which belongs to the category of a sparse matrix, and its weight can be defined in the following two ways:

(1) Thermonuclear definition
  (11) $$\begin{array}{c} W_{ij}=\left\{\begin{array}{cc} e^{-\left({\left\|x_{i}-x_{j}\right\|}^{2}/t\right)}\text{,} & ifx_{j}\in N\left(x_{i}\right)\text{,}\\ 0\text{,} & otherwise\text{,} \end{array}\right. \end{array}$$
where N(xi) represents the vectors of all neighbors.
(2) Simplified definition:

If the vector between xi and xj, it is Wij = 1; otherwise, it is Wij = 0. Among them, Wij is set to 1 so that the similarity of the original data in the mapped hash code is close. Assuming that V is a set of transformation vectors, the objective function is simplified to

(12) $$\begin{array}{c} {\sum_{i,j}\left(y_{i}-y_{j}\right)}^{2}W_{ij}={\sum_{i,j}\left(v^{T}x_{i}-v^{T}x_{j}\right)}^{2}W_{ij}\\ =2\sum_{i}v^{T}x_{i}D_{ii}x_{i}^{T}v-\sum_{ij}v^{T}x_{i}W_{ij}x_{i}^{T}v\\ =2v^{T}X\left(D-W\right)X^{T}v\\ =2v^{T}XLX^{T}v\text{,} \end{array}$$

where *D* is the diagonal matrix and *L* is the Laplacian matrix, *L* = D – W. The larger the Di, the more important the corresponding Yi, so add a restriction.

(13) $$\begin{array}{c} Y^{T}DY=1\Rightarrow v^{T}XDX^{T}v=1\text{.} \end{array}$$

Minimizing the objective function can be expressed as follows:

(14) $$\begin{array}{c} \begin{array}{c} arg_{v^{T}XDX_{v=1}^{T\min}}v^{T}XLX^{T}v\text{,}\\ XLX^{T}v=\lambda XDX^{T}v\text{.} \end{array} \end{array}$$

## 4. Probabilistic Leaker Judgment Scheme Based on the Trust Model

### 4.1. Trust Model in Social Networks

Trust is subjective, transferable, and asymmetric. It can be understood as “a person's subjective expectation of another person in the future,” which promotes the exchange of information between social network users. Therefore, in the relevant content, the degree of trust between nodes is regarded as one of the important factors of whether they will spread messages between them. The credibility is based on the user's past credibility performance. Therefore, in this section, we will focus on the calculation of trust between neighboring users.

Many users are unwilling to publicly judge the trust level of neighbor users in social networks. In most platforms, the relationship between two points is two-way and can only be established after confirmation by both parties, such as Facebook and WeChat. But, in other platforms, the node relationship is not bidirectional, and only part can be changed under the premise of mutual attention. Regardless of whether or not, the trust between them is directional but asymmetric. Secondly, the relevant definition and calculation formula of the trust model are proposed. Finally, we will show how to build a trusting social network.

#### 4.1.1. Related Definitions

**Definition 1 .**

User similarity: It describes the similarity of attributes and interests among users.

Many studies have proposed similar concepts to express the similarity between objects. The similarity between user Xi and user xj is represented by Sim(Xi, xj).

**Definition 2 .**

User interaction: It depicts information that two adjacent users have exchanged before.

The historical interaction information between users has an important influence on the degree of trust between users, such as the frequency of interaction, the number of interactions, and so on. The trust score of interaction between users is expressed as Int(Xi, xj).

**Definition 3 .**

Network structure: important structure information between social node pairs. Depicts the influence of the topology map on the trust degree, and the trust value calculated by the social network structure is expressed as NS(ui, uj).

#### 4.1.2. Trust Calculation Model

The trust between all adjacent users is initially equal, and the trust value we evaluate is represented by any two directly connected users in an asymmetric social network T(ui, uj). The comprehensive trust value uj of the user interface is based on the similarity between users. The calculation formula of T(UI, uj) is as follows:

(15) $$\begin{array}{c} T\left(u_{i},u_{j}\right)=\alpha \cdot Sim\left(u_{i},u_{j}\right)+\beta \cdot Int\left(u_{i},u_{j}\right)+\gamma \cdot NS\left(u_{i},u_{j}\right)\text{,} \end{array}$$

where the values of T(ui, uj), Sim(ui, uj), Int(ui, uj), and NS(ui, uj) are all in the range of 0 to 1.0 means that user ui does not trust user uj at all, that is to say, T(ui, uj) = 1 means full trust, and the larger the value, the higher the trust. The adjustment of the value of *α*, *β*, and *γ* will make the trust model to be optimized along a specific dimension. The attributes in the social network determine the distribution of the specified weight.

We choose factors that have a great influence on the application, not all factors. Next, we will describe the calculation of three important factors affecting trust, in order:

(1) Similarity calculation: The similarity between users in the model includes interest similarity, as well as similarity of different attributes, such as gender, age, educational background, and social background. It is easier to trust each other with similar attributes than without similar attributes. The same is true for similar collaborative filtering algorithms. The calculation formula for the similarity between users is as follows:
  (16) $$\begin{array}{c} Sim\left(u_{i},u_{j}\right)=w_{1}f\left(A_{u_{i}1},A_{u_{j}1}\right)+w_{2}f\left(A_{u_{i}2},A_{u_{j}2}\right)+\cdots +wnf\left(A_{u_{i}n},A_{u_{j}n}\right)\text{,} \end{array}$$
where *n* is the number of attributes available in the network and wk is the weight of the similarity between the attributes of user ui and the attributes of user uj, and the value range is 0 to 1. The larger the value, the greater the similarity of the attribute.
The last three formulas in Table 1 are used to calculate the similarity of multivalued attributes. Table 1 lists the user attribute information obtained by using the appropriate similarity calculation formula. Single-valued attributes are calculated by simple comparison and interval ratio.
(2) User interaction computing: a basic feature in social networks. The more interaction between users, the higher the degree of trust between them, and they will think each other is more trustworthy.
  (17) $$\begin{array}{c} Int\left(u_{i},u_{j}\right)=\frac{\left|A\left(u_{i},u_{j}\right)\right|}{\sum_{u_{j}\in N}A\left(u_{i},u_{j}\right)}\text{,} \end{array}$$
where A (ui, uj) represents the total number of interactions between user ui and user uj, and N is the user's neighbor set. The essence of formula (20) is the ratio of the number of interactions between user ui and user uj to the total number of interactions of user ui.
(3) Social network structure. The structure of a social network can be expressed as N(G, E), where *G* represents the set of user nodes and *E* represents the edge of the relationship between users.
  (18) $$\begin{array}{c} NS\left(u_{i},u_{j}\right)=\frac{\left(\left|\Gamma \left(u_{i}\right)\cap \Gamma \left(u_{j}\right)\right|\right)+\left(\left|C\left(u_{i}\right)\cap C\left(u_{j}\right)\right|\right)}{\left(\left|\Gamma \left(u_{i}\right)\cup \Gamma \left(u_{j}\right)\right|\right)+\left(\left|C\left(u_{i}\right)\cup C\left(u_{j}\right)\right|\right)}\text{.} \end{array}$$

Calculate the trust between users based on the social network structure, by calculating the mutual friends between users, the user's entry degree (the number of edges pointing to the user), and the exit degree (the number of edges pointing to other nodes). The more mutual friends a user has, the more likely they are to trust each other. The rule of “a common friend is equal to a common neighbor” is also applicable to social networks. After the area is divided, the more common communities owned by users, the higher the degree of understanding. The relationship structure between users is constantly changing with the dynamic network. The interaction history and hobbies between adjacent users are also constantly changing, so the trust model should be updated regularly.

The trust calculation scheme proposed above is a basic algorithm that can be adjusted to optimize the results of any given network. In fact, because trust is a relatively vague concept, it will be implemented in different ways in the network environment and community environment, so it is unreasonable to apply a set of strict algorithms to all networks. When implementing the algorithm in the network, we should understand the basic characteristics of the network and the acquired data resource information, so as to adjust the implementation of the parameters accordingly. In the following content, we can use the trust value and user credibility to determine the probability of a certain user in a network leakage event.

In fields such as e-commerce, it is often necessary to rate interactions to quantify the credibility of Facebook users. The reputation value in the model of this article is an important factor that affects users' unauthorized communication. In addition, there are more complex evaluation systems. Therefore, we formally give a conceptual definition of reputation.

(19) $$\begin{array}{c} Rp\left(u_{i}\right)=\frac{1}{n}\sum_{u_{j}\in N\left(u_{i}\right)}T\left(u_{j},u_{i}\right)\text{,} \end{array}$$

where N(ui) represents the neighbor set of user ui, and *n* is the number of users in the N(ui) set.

### 4.2. The Leaker's Judgment Plan

There are edges between two nodes. The definition of social network topology indicates that they have interacted before and have a higher probability of interaction in the future. In addition, user credibility is also an important factor that affects whether users are willing to disclose information. The publisher-centered information dissemination probability model is based on the weighted trust and reputation social network topology between the trust attributes and the node reputation attributes and calculates the probability of illegal information dissemination for each recipient.

As shown in Figure 2, the user publishes a piece of digital media to the recipient. When digital media is found on the public platform, the user hopes to find the person responsible for the leak. The method proposed in this chapter is to calculate the probability of a user being a recipient of disclosure based on the social attributes in the social network. Figure 2 defines a G-weighted social network topology (the total number of nodes is W). We choose a path of no more than three hops under two factors: first, in reality, more than three hops are less spread; second, the number of users leads to an explosive increase in the computational complexity of each hop.

Build a smaller network topology, including necessary nodes, and reduce the time complexity of path search.  Figure 3 is the initial structure of the social network.  Figure 4 is a common topology of a small social network. As shown in Figure 4, the first-level nodes are the direct friends of user *D*; the second-level nodes are the friends of user D's direct friends; and so on. As shown in Figure 4, we have established node *D* of the nearest neighbor extension GD. The *D* node can be a user group or user solves U. By three-hop nearest neighbor set intersection extension user set *R* and three-hop nearest neighbor set extension for user U, we can get the network topology of all nodes and can spread information, which we call *G*.

After obtaining the social network topology G' for the search of information propagation paths, we use the DFS method of depth-first search to obtain all paths between two nodes that are less than three hops. Assume that nodes B, K, P, *Q*, and V belong to the receiver user set RI, node N is the message publisher, and node *D* is the unauthorized information receiver U. Then we found all the paths from the user setting RI to unauthorized user U, as shown in Table 2. At this point, we have all possible paths within three hops from the receiving user set Ri to the unauthorized user U (i.e., all message propagation paths). Table 2 just shows a simple idealized example, illustrating that the topology of a real social network is very complicated.

The edge weight W(ni,nj) in the topological graph of Figure 4 represents the probability of the user spreading information. The factors that affect the probability of information dissemination include the degree of trust among users and the credibility of the information. The credibility of information is essentially an important criterion for reflecting whether users will spread information about others without authorization. If there is a directed edge between two nodes, the edge weight W(Ni, Nj) can be calculated by the following formula (similarly, W(Ni, Nj) can be calculated):

(20) $$\begin{array}{c} W\left(N_{i},N_{j}\right)=\left\{\begin{array}{c} \frac{T\left(N_{i},N_{j}\right)}{Rp\left(N_{i}\right)},if\;T\left(N_{i},N_{j}\right)<Rp\left(N_{i}\right)\text{,}\\ T\left(N_{i},N_{j}\right),if\;T\left(N_{i},N_{j}\right)\geq Rp\left(N_{i}\right)\text{.} \end{array}\right. \end{array}$$

When we find a copy of the leaked information, we can directly lock the uploader A of the copy. Transform the problem. In particular, if A is a user in the RI, the leaker can be directly identified. When A is not a member of RI, we perform the following steps to identify the leaker. First, we traverse the social network topology G′=(N′, E′) to find all the paths of the target user *u*; these paths do not include any other users in the receiver set except Ri.

(21) $$\begin{array}{c} W_{j}\left(R_{i},U\right)=\left\{\begin{array}{c} W\left(R_{i},N_{x}\right)\times W\left(N_{x},N_{y}\right)\times W\left(N_{y},U\right)if\;length\left(l_{ij}\right)==3,\\ W\left(R_{i},N_{k}\right)\times W\left(N_{k},U\right)if\;length\left(l_{ij}\right)==2\left(3-7\right),\\ W\left(R_{i},U\right)if\;length\left(l_{ij}\right)==1\text{.} \end{array}\right. \end{array}$$

By comparing the values of all paths Wj(Rj, U) from Ri to the target user U, the path with the largest weight is found and defined as the weight from the user Ri to the target user U, namely

(22) $$\begin{array}{c} W\left(R_{i},U\right)=\mathrm{MAX}\left\{W_{j}\left(R_{i},U\right)\left|j\in N*\right.\right\}\text{.} \end{array}$$

Before judging, we should determine which paths are reasonable, so we define a threshold *M* that is the average of all information propagation paths. When a certain information propagation path is greater than *M*, it indicates that the path is reasonable, so

(23) $$\begin{array}{c} W*\left[R_{i},U\right]=\left\{\begin{array}{c} W\left(R_{i},U\right),\mathrm{if}\;W\left(R_{i},U\right)\geq M,\\ 0,if\;W\left(R_{i},U\right)<M\text{.} \end{array}\right. \end{array}$$

After all the propagation paths are obtained, the probability of a certain user's leakage is obtained by

(24) $$\begin{array}{c} \mathrm{Pr}\;*\left(R_{i},U\right)=\frac{W*\left(R_{i},U\right)}{\sum_{i\in \left[1,n\right]}\left(R_{i},U\right)}\text{,} \end{array}$$

where Pr ∗ (Ri,U) is the probability of user Ri leaking information.

The judgment algorithm is realized by MATLAB programming. In order to verify the accuracy of the algorithm, we chose the Facebook data set downloaded from the Snap website. The data set contains a total of 4,034 nodes and 88,434 edges. In order to verify the accuracy of the leakage probability judgment algorithm, we can only manually calculate the path between nodes that are less than or equal to two hops. By comparing the leakage probability judgment algorithm to calculate the result of user leakage probability and the result of statistical user manual leakage probability, the accuracy of the algorithm is obtained. At the same time, we calculated the time cost of the leak probability judgment algorithm within 3 hops of 10 pairs of nodes, as shown in Table 3. It can be seen from the table that the accuracy of the user leakage probability algorithm can reach 100%, and the time cost is within an acceptable range.

## 5. Deterministic Leaker Tracking Scheme Based on Digital Fingerprints

### 5.1. System Model

Digital fingerprints can effectively solve the increasingly concerned digital copyright issue. Therefore, the research on digital fingerprints is of great significance. At present, there are two main research directions for digital fingerprints: one is the information (such as text) itself, which uses algorithmic information to get a fingerprint. When it is found that the fingerprint generated by a suspicious leak is the same as the suspicious version, then a similar method is used to judge whether there is plagiarism between documents. The other is to obtain a digital fingerprint through the field of digital copyright and incorporate it into digital media technology to track leakers. The fingerprint here is a non-specific fingerprint, which is a binary sequence added in the form of a digital watermark. Every digital media purchased by consumers has a unique digital fingerprint. When piracy occurs, it can be traced back to the source of the leak accurately. Compared with traditional digital fingerprints, the differences between digital fingerprints in social networks are as follows.

Traditional digital fingerprint coding can even be applied to more than one million users, but it is ahead of the user level of social platforms. Therefore, the existing digital fingerprint coding cannot provide the uniqueness of fingerprint codes for such a large number of user networks. The fingerprint identification system not only embeds fingerprints into multimedia content but also has a series of codes and corresponding tracking algorithms for identity traitors. The basic system model of the digital fingerprint tracking scheme is shown in Figure 5. The publisher sends the information *Z* to each recipient, which includes many versions of different types of information. If illegally copied information is detected, the leaker can be identified by the difference in fingerprints. Input a code word w' and output at least one leaker, so traditional digital fingerprint coding is not suitable for digital fingerprint coding in social networks.

### 5.2. Digital Fingerprint Detection and Simulation Results and Analysis

Hash BF digital fingerprint coding scheme still has a challenging and urgent problem: the large-scale fingerprint set makes fingerprint detection and tracking very difficult or even impossible. However, it is still an arduous task to distinguish the distance between fingerprints of all users using the traditional linear search method. The digital fingerprint code word proposed in this paper is a binary sequence. Compared with the traditional high-dimensional data search, the efficiency is extremely low, and the efficiency and accuracy are further improved. We build an index table based on the user's digital fingerprint and user ID. The format of the index table is shown in Table 4, where the hash codes are sorted. For the hash code sorting index table, dichotomy can be used to quickly find the nearest neighbor set of the target user's hash code. We can appropriately expand the search range and search the user ID and complete fingerprint sequence in the obtained nearest neighbors.

Search the binary index table to find the closest hash code and extract the corresponding fingerprint and user identifier. The specific process is to compare each user's fingerprint with the nearest target fingerprint. The user with the smallest distance is considered to be the culprit. Convert table content into image content; the image is shown in Figure 6:.

1. In order to verify the feasibility and performance of the Hash BF fingerprint allocation algorithm, we downloaded three sets of social media data from the Stanford University SNAP1 website for simulation experiments, namely Facebook, Twitter, and Google+. The content of the data set is formatted as a TXT file, which contains the nodes in the social network and the edges between nodes. The former is not directed, and the latter two are directed. The specific data set size is shown in Table 5.
2. In order to verify the performance of the GLPP algorithm in maintaining the structural characteristics of the social network, a twofold cross-validation method is used for experiments.
3. We use DCT intermediate frequency digital algorithm and its corresponding Filipe extraction algorithm to verify the accuracy of the Hash BF algorithm in actual fingerprint scenes and conduct diving and fingerprint code extraction experiments. After extracting the fingerprint from the suspicious copy, the fingerprint is divided into two parts: hash code and binary random sequence code. Then we compare the distance between Hamming and the user's hash code to find all the neighbors closest to the whistleblower. The calculation methods of accuracy and recall are as follows:

(25) $$\begin{array}{c} \left\{\begin{array}{c} precision=TP\left(TP+FP\right),\\ recall=TP\left(TP+FN\right). \end{array}\right. \end{array}$$

So far, we have only maintained the nearest neighbor performance of our algorithm under different *d* values. In order to show the performance advantages of our algorithm over other classic algorithms, we also selected the Twitter data set in the experiment and set the *d* value to 0.

Traditional privacy research has not kept pace with the times. The scheme introduced in this article first searches the nearest neighbor set and then searches the nearest neighbor set according to the binary random sequence code. The specific process is to compare each user's fingerprint with the Hamming distance of the target fingerprint in the nearest neighbor set. The user with the smallest Hamming distance is judged as a leaker. In our Google+ social network collection, we randomly select from 10,000 to 100,000 nodes for the experiment, where we selected 10 times the threshold, Hamming distance d=3, and hash code and binary random sequence code length of 64 bits.

## 6. Conclusion

In online social networks, the traditional research on privacy protection is mainly to prevent information from being intercepted by intruders during transmission. This can be achieved by implementing multiple encryption methods. Probabilistic judgment based on trust is the most commonly used privacy protection method for information leakage. With the continuous development of the Internet age, the speed of information dissemination has also increased, and many people have applied anonymization and differential algorithms to protect their privacy. However, few people study or write articles on common leakage methods. Perhaps it is too common. Most people do not have the confidence to find a way to crack or prevent information leakage. In the real world, if a publisher publishes digital content on a certain platform, then the user who receives the content may be one person or multiple people because, once the information is disclosed, it is equivalent to being placed. In the eyes of many people in society, everyone can see, so the data cannot be protected. Once users publish digital content (assuming that private information is not invaded by intruders), if unauthorized information is detected to be spread, the source of the leakage must be traced. So far, many privacy protection methods including differential protection algorithms, encryption algorithms, access control strategies, and anonymization have been researched and applied. This article also introduces the trust degree model and the encryption protection of private information, hash mapping, and digital fingerprint algorithms and uses the several methods mentioned in the former, and constructs a weighted social network topology based on trust on the premise of several methods mentioned previously. The shortest path algorithm is backed by the calculation probability, and an information release system for user security classification and information sensitivity classification has been established. With an attitude that can reduce the risk of information leakage and maintain the security of private information, a comprehensive system has been developed and improved; thereby, it can effectively reduce the risk of user information being leaked. While ensuring that user information is not leaked, it can also ensure the normal operation of the online social system so that the interests of online social users are protected. The system solves the urgent need for online social network users and platforms, also blocks the illegal path of bad elements, and promotes the operation and development of the network social system on a normal track.

## Figures and Tables

**Figure 1:** Social network model.

**Figure 2:** Information disclosure model weighted by trust and honor.

**Figure 3:** Initial structure of the social network.

**Figure 4:** Layered network topology diagram.

**Figure 5:** Digital fingerprint scheme system model.

**Figure 6:** Information leakage tracking flowchart.

**Table 1:** Similarity calculation method.

Calculation	Formula	Description
Simple comparison	S(ui, uj) = 1, if x＝y 0, if x≠	x and *y* are the attributes of user ui and uj, respectively
Interval ratio	S(ui, uj) = 1-|x-y|/N	N can be max(|x-y) or manually set
Jaccard coefficient	J(ui, uj) = |*A*(*u*i)∩*A*(*uj*)|/|*A*(*u*i) ∪ *A*(*uj*)|	A(ui) and A(uj) are the attribute sets of user ui and uj, respectively
Cosine similarity	Cos(ui, uj) = |*V*(*u*i)∩*U*(*uj*)|/‖*V*(*u*i)‖‖V(*uj*)‖	The vectors V(ui) and V(uj) are the attributes of user ui and uj, respectively
Pearson coefficient	P(ui,uj) = $\sum_{k=1}^{n}\left(xk-\bar{x}\right)\left(yk-\bar{y}\right)/\sqrt{\sum_{k=1}^{n}\left(xk-\bar{x}\right)}\sqrt{\sum_{k=1}^{n}\left(yk-\bar{y}\right)}$	xk and yk represent different attributes of user ui and uj, respectively

**Table 2:** Summary of paths within three hops.

	Path 1	Path 2	Path 3	Path 4
Node B	B—D	B—C—D	B—A—C—D	No
Node K	K—D	K—F—D	K—I—F—D	K—H—E—D
Node P	No	No	No	No
Node Q	Q—C—D	Q—C—B—D	No	No
Node V	V—u—B—D	V—A—B—D	V—A—C—D	No

**Table 3:** The accuracy and time cost of the algorithm for judging the probability of leakage.

Node pair	1	2	3	4	5	6	7	8	9	10
Accuracy	100%	100%	100%	100%	100%	100%	100%	100%	100%	100%
Time overhead (ms)	20,993	37,012	76,505	41,345	10,965	19,688	20,675	11,587	50,049	26,673

**Table 4:** Digital fingerprint index table.

Hash code (ordered)	Random sequence code	User ID
0x2DF3C9EA	0xAFB68CD7	94………………vv
0x2DF3C9EA	OxFB6EE3D7	Kk………………66
0x2DF3C9EB	0xAD68CD7F	Hk………………ki
0xFFE2A97 C	0xAFB64CD7	54………………gr
0xFFE2A97D	OxBF6E8AD7	Rt………………6g

**Table 5:** Social network data set attributes.

Data set	Number of nodes	Number of edges	Do you want to report back?	Number of communities
Facebook	4,039	88,234	No	10
Twitter	81,306	1,768,149	Yes	1,000
Google+	107,614	13,673,453	Yes	133

## Data Availability

The data used to support the findings of this study are available from the corresponding author upon request.
